RETRACTED

# Regulation of Cigarette Smoke (CS)-Induced Autophagy by Nrf2

**DOI:** 10.1371/journal.pone.0055695

**Published:** 2013-04-09

**Authors:** Lingxiang Zhu, Erika C. Barret, Yuxue Xu, Zuguo Liu, Aditya Manoharan, Yin Chen

**Affiliations:** 1 Department of Pharmacology and Toxicology, University of Arizona, Tucson, Arizona, United States of America; 2 School of Medicine, Xiamen University, Xiamen, China; National Jewish Health, United States of America

## Abstract

Cigarette smoke (CS) has been reported to induce autophagy in airway epithelial cells. The subsequent autophagic cell death has been proposed to play an important pathogenic role in chronic obstructive pulmonary disease (COPD); however, the underlying molecular mechanism is not entirely clear. Using CS extract (CSE) as a surrogate for CS, we found that it markedly increased the expressions of both LC3B-I and LC3B-II as well as autophagosomes in airway epithelial cells. This is in contrast to the common autophagy inducer (i.e., starvation) that increases LC3B-II but reduces LC3B-I. Further studies indicate that CSE regulated LC3B at transcriptional and post-translational levels. In addition, CSE, but not starvation, activated Nrf2-mediated adaptive response. Increase of cellular Nrf2 by either Nrf2 overexpression or the knockdown of Keap1 (an Nrf2 inhibitor) significantly repressed CSE-induced LC3B-I and II as well as autophagosomes. Supplement of NAC (a GSH precursor) or GSH recapitulated the effect of Nrf2, suggesting the increase of cellular GSH level is responsible for Nrf2 effect on LC3B and autophagosome. Interestingly, neither Nrf2 activation nor GSH supplement could restore the repressed activities of mTOR or its downstream effctor-S6K. Thus, the Nrf2-dependent autophagy-suppression was not due to the re-activation of mTOR-the master repressor of autophagy. To search for the downstream effector of Nrf2 on LC3B and autophagosome, we tested Nrf2-dependent genes (i.e., NQO1 and P62) that are also increased by CSE treatment. We found that P62, but not NQO1, could mimic the effect of Nrf2 activation by repressing LC3B expression. Thus, Nrf2->P62 appears to play an important role in the regulation of CSE-induced LC3B and autophagosome.

## Introduction

Autophagy is a regulated catabolic process, by which cellular components are sequestered in the vesicular system and later delivered to lysosomes for degradation and recycling of biogenic components [1]. Autophagy has been demonstrated to play a critical role in maintenance of cellular homeostasis and the adaption to environmental stress such as oxidative stress, starvation, hypoxia and infection [1]–[4]. The final outcome of autophagy could be either cell death or survival, and its morphological and biomedical features are distinct from other cell death pathway (e.g. apoptosis). A set of autophagy-related genes (ATG) have been identified to be responsible for the regulation of each step of autophagic pathway [5].

RETRACTED

Most of the ATG proteins are highly conserved in mammals. Class III phosphoinositide 3-kinase (PI3K) and ATG6 initiate the formation of autophagosomes. Furthermore, two ubiquitination-like conjugation systems are required for autophagosome formation. One of these systems mediates the conjugation of ATG12 to ATG5 [6], and the other mediates a covalent linkage between LC3B (Atg8) and phosphatidylethanolamine (PE) [7]. An ATG12-ATG5 conjugate is present on the outer side of the isolation membrane and is required for elongation of the isolation membrane [8]. A PE-conjugated form of LC3B localizes on the isolation membrane and the autophagosome membrane [9], [10]. The unconjugated (designated as LC3B-I) and conjugated forms (designated as LC3B-II) of LC3B can be easily separated by SDS-PAGE and detected by antibody staining on the western blot [11]. The intracellular LC3B-II can usually be recognized by its unique “punctate dot” structure [9], [11]when the cells are transfected with GFP-LC3B and challenged with autophagy-inducers. Because the level of LC3B-II is generally correlated with the number of autophagosomes [9], the currently established standard [12] uses the amount of LC3B-II (through either *in vitro* western blot or *in vivo* punctate formation) as the hallmark and surrogate for autophagic activity.

Despite the overwhelming studies on autophagy in diseases, very few have been carried on non-malignant airway diseases. Recently, several studies have demonstrated that cigarette smoke (CS) or cigarette smoke extract (CSE) induces autophagy in lung cells [13]–[15], and this autophagic process appears to play a critical role in the pathogenesis of emphysema [13], [16]. In these studies, reactive oxygen species (ROS) has been suggested to mediate CSE-induced autophagy, but the detailed mechanism is not entirely clear. Interestingly, it is well established that anti-oxidant systems such as Nrf2 protect the animal from CS-induced lung injury and airway inflammation [17], and the deregulation of Nrf2 contributes to the pathogenesis of emphysema [18]–[20]. Thus, we speculate that Nrf2 may also have the ability to regulate autophagy in CS/CSE exposure model.

## Materials and Methods

### 1. Chemicals, antibodies, and plasmids

3-Methyladenine (3-MA), E64D, Pepstatin A were purchased from Sigma-Aldrich (St. Louis, MO). Antibodies against LC3B, p62 and HO-1 were from MBL International (Woburn, MA). Nrf2, Keap1 and Actin antibodies were purchased from Santa Cruz Biotechnology (Santa Cruz, CA). Antibodies against p-mTOR (Ser 2448) and p-S6K (Thr 389) were purchased from Cell signaling technology (Danvers, MA). The plasmids of Nrf2 and GFP-LC3B were kind gifts from Dr. Jingbo Pi (The Hamner Institutes, RTP, NC) and Dr. Tamotsu Yoshimori (Osaka University, Osaka, Japan), respectively. P62 plasmid and two ARE-reporters (pARE_Gst-luc contains ARE sequence from mouse glutathione S-transferase Ya subunit promoter [21]; pARE_NQO1-luc contains ARE sequence from human NQO1 promoter [22]) were kind gifts from Dr. Donna Zhang (University of Arizona, AZ).

RETRACTED

### 2. Cell culture

BEAS-2B was cultivated on regular tissue culture dish in a humidified atmosphere of 5% CO_2_/balanced air at 37°C as described before [23]. Before experiments, the cells were cultivated in growth factor free medium for 16 hrs.

### 3. CSE preparation and treatment

CSE preparation was based on the protocol described previously with some modifications [15]. Briefly, Kentucky 1R3F research-reference filtered cigarettes (The Tobacco Research Institute, University of Kentucky, Lexington, Kentucky) were smoked using a peristaltic pump (VWR International). Cigarette smoke from three cigarettes was bubbled through 30 ml of F12 medium. This solution was regarded as 100% strength CSE. pH was adjusted to 7.4 and used within 20 min after preparation. For the treatment, CSE was diluted directly into the culture medium for the indicated percentage.

### 4. Transient transfection and dual luciferase reporter assay

For the dual-luciferase reporter gene assay, BEAS-2B cells were transfected with the pARE_Gst-luc or pARE_NQO1-luc along with the Renilla luciferase expression plasmid pGL4.74 (hRluc/TK) (Promega). At 24 hrs post-transfection, the transfected cells were treated with CSE for 24 hrs or immersed in the starve media for 6 hrs. Then, the cells were lysed with passive lysis buffer (Promega) and both firefly and Renilla luciferase activities were measured with the dual-luciferase reporter assay system purchased from Promega. Firefly luciferase activity was normalized to Renilla luciferase activity. The experiment was carried out in triplicate and expressed as the mean ± the standard deviation (SD).

### 5. Live imaging of autophagosome

BEAS-2B cells were transfected with GFP-LC3B. At 24 hrs post-transfection, the cells were treated with or without CSE for 24 hrs. Fluorescence Images were acquired by using of a confocal microscope (LSM 510 meta, Carl Zeiss, Thornwood, NY). Six random areas (20X) were selected for the quantification on each slide, and triplicate samples were included for each experimental group. Cells containing “punctate dot” were counted and expressed as percentage of the total cells.

RETRACTED

### 6. Western blot

Total cellular proteins were collected and western blot analysis were performed based on the methods described previously [24]. The sources of antibodies have been described in the “Chemicals, antibodies, and plasmids”. Equal protein load was confirmed using the staining of anti – actin antibody.

### 7. Real-time PCR

Real-time PCR was performed as described previously [25]. cDNA was prepared from 3 µg of total RNA with Moloney murine leukemia virus (MoMLV)–reverse transcriptase (Promega, Inc.) by oligo-dT primers for 90 min at 42°C in a 20-µl reaction solution, and was then further diluted to 100 µl with water for the following procedures. Two microliters of diluted cDNA were analyzed using 2x SYBR Green PCR Master Mix by an ABI 5700 or ABI Prism 7900HT Sequence Detection System (Applied Biosystems Inc., Foster City, CA), following the manufacturer's protocol. Primers (Table 1) were used at 0.2 µM. The PCR reaction was performed in 96-well optical reaction plates, and each well contained a 50-µl reaction mixture. The SYBR green dye was measured at 530 nm during the extension phase. The relative mRNA amount in each sample was calculated based on the ΔΔC_t_ method using housekeeping gene *GAPDH*. The purity of amplified product was determined from a single peak of a dissociation curve. Efficiency curves were performed for each gene of interest relative to the housekeeping gene, based on the manufacturer's instructions. Results were calculated as fold induction over control, as described previously [25].

**Table 1:** Realtime Primers.

Gene	Primers	
LC3B	forward	AGAGCAGCATCCAACCAAAAT
	reverse	TGAGCTGTAAGCGCCTTCTAA
GAPDH	forward	CAATGACCCCTTCATTGACC
	reverse	GACAAGCTTCCCGTTCTCAG

### 8. Small interference RNA (siRNA) and transient transfection

Two different siRNAs were used for the knockdown of each gene. siRNA targeting Nrf2 (#1: GTAAGAAGCCAGATGTTAA) [26], #2: AAGAGTATGAGCTGGAAAAAC [27]), Keap1 (#1: GGGCGTGGCTGTCCTCAAT) [26], #2: TGAACGGTGCTGTCATGTA [28]) NQO1 (#1: GGACATCACAGGTAAACTG, #2: GAACCTCAACTGACATATA [29]) and P62 (#1: GCATTGAAGTTGATATCGA) [30]) were synthesized by Ambion (Austin, TX). The second set of P62 was the pooled siRNA purchased from Santa Cruz Biotechnology (Santa Cruz, CA). Since the results were identical, only the data from #1 were presented. In addition, non-targeted control siRNA (siRNA #1 from Ambion) and individual randomized sequence for Nrf2, Keap1, NQO1 and P62 were also tested as described in the previous publication [31]. Because of identical results, only siRNA #1 was used as control for all the siRNA knockdown studies. siRNA was transfected into cells using lipofectamine^TM^ 2000 (Invitrogen, Carlsbad, CA) based on manufacturer's instruction. Successful knockdown of the target was confirmed by realtime RT-PCR and western blot.

RETRACTED

### 9. Measurement of Intracellular Reactive Oxygen Species by Live Cell Imaging

Reactive oxygen species (ROS) production was determined using chloromethyl-2′,7′-dichlorodihydrofluorescein diacetate (CM-H_2_DCFDA; Molecular Probes, Eugene, OR) according to the manufacturer's instruction. Briefly, cells were rinsed twice with warm phenol red-free medium and then loaded for 30 min with CM-H_2_DCFDA (3 μM) in medium without phenol red. The cells were rinsed three times for removal of the extracellular dye, and the medium was replaced with phenol red-free medium. Then the cells were loaded into a live cell imaging incubator (Carl Zeiss, Thornwood, NY) at 37°C in a 5% CO_2_ atmosphere. Live cell images were continuously recorded before and after CSE treatment by confocal microscopy (LSM 510 meta, Carl Zeiss).

### 10. Statistical analysis

Experimental groups were compared using a two-sided Student's *t* test, with significance level set as *P*<0.05. When data were not distributed normally, significance was assessed with the Wilcoxon matched-pairs signed-ranks test, and *P*<0.05 was considered to be significant. Matlab 6.0 with statistics toolbox (MathWorks, Inc., Natick, MA) was used for analyses of the data.

## Results

### 1. CSE induced LC3B-I and II as well as autophagosomes, but CSE-induced autophagy was different from that induced by starvation

Starvation-induced autophagy has been extensively studied. Recently, CSE has also been shown to induce autophagy in airway cells [13]–[15]. The hallmark of autophagy is the elevation of LC3B-II [12]. We compared these two stimuli in the induction of autophagy in airway epithelial cells. Indeed, both starvation and CSE dramatically increased cellular autophagosomes as compared with non-treated control (Fig. 1A). Significant increase of LC3B-II and decrease of LC3B-I, thus the increase of LC3B-II: LC3B-I ratio, was observed in the starved cells at both 2 hrs and 6 hrs (Fig. 1B). This conversion (from LC3B-I to LC3B-II) was significantly blocked by 3-MA (type III PI3K kinase inhibitor) treatment, suggesting that a classical autophagy dependent mechanism is responsible for this process. Starvation for 24 hrs caused significant cell death and the reduction of overall LC3B in these cells (data not shown). Thus, we did not include this time point. Different from starvation, CSE increased both LC3B-I and LC3B-II time- and dose-dependently (Fig. 1C). At lower dose (4%), CSE treatment slightly induced both LCB-I and II level; but at the higher dose (10%), LCB-I and II were elevated at 6 hrs and markedly increased at 24 hrs. CSE also increased the level of Nrf2 (Fig. 1C), a master regulator of cellular antioxidant response. Nrf2 appeared to be elevated early (6 hrs) and later slightly subsided (24 hrs). Consistent with Nrf2 increase, the activities of two different ARE reporters (pARE_Gst-luc or pARE_NQO1-luc) were significantly increased in CSE treated as compared with non-treated controls (Fig. 1D). The highest dose (i.e. 20%) appeared to cause outright toxic effects that shut down all the processes. Thus, we used 10% CSE for the following studies. In contrast, starvation had no effect on Nrf2 (Fig. 1B) or ARE promoter activities (Fig. 1D).

RETRACTED

**Figure 1:** CSE-enhanced autophagy is different from the starvation-induced autophagy in airway epithelial cells. All western blot images were the representative image from at least three independent analyses, and Actin was use as a loading control. A) Increase of cellular autophagosome by live imaging. Cells stably transfected with GFP-LC3B were treated either with 10% CSE for 24 hrs or were immersed in HBSS buffer (starvation or S) for 6 hrs. Control (C) was sham (medium)-treated sample. Live images were recorded. “punctate dots” of GFP-LC3B were the indication of autophagosomes. B) Starvation induced autophagy but not Nrf2. Cells were immersed in HBSS (S) without or with 3-Methyladenine (3-MA). Total protein was collected at the indicated time point and subject to western blot analysis. C) CSE induced both autophagy and Nrf2. Cells were treated with different dose (as indicated in the figure) for either 6 hrs or 24 hrs. Total protein was collected and subject to western analysis. D) CSE induced ARE-reporter activation. Two different ARE-reporters were transfected into cells. 24 hrs later, the cells were treated with 10% CSE for 24 hrs or immersed in HBSS (S) for 6 hrs. Cell lysates were prepared and subject to dual luciferase assay. Relative luciferase unit (RLU) was calculated as described in the Materials and Methods. Fold induction  =  RLU of treated cells/RLU of control cells. *: p<0.05, n = 5. NS: not significant.

### 2. CSE regulated LC3B-I and II at transcriptional and post-translational levels

Since LC3B is the critical player of autophagy and its dynamics in CSE treated cells were clearly different from the classical autophagy inducer-starvation, we examined the potential molecular mechanism underlying CSE-induced LC3B-I and II. As shown in Fig. 2A, CSE increased LC3B-I as early as 1 hrs; but only starting at 6 hrs, LC3B-II was elevated. As comparison, Nrf2 induction by CSE peaked at 6 hrs and decreased at 24 hrs. By realtime PCR, we found that LC3B mRNA was moderately (but significantly) increased (Fig. 2B). Since LC3B is known to be degraded in the lysosomal compartment after the fusion between autophagosome and lysosome, we asked the question whether or not the elevation of LC3B protein by CSE was perhaps caused by the blockade of this process. LC3B-I was not changed (or slightly increased) either by the blockade of lysosomal protease activity via the treatment of E64D + pepstatin A (two common lysosomal inhibitors), or by the inhibition of autophagosome formation using 3-MA (Fig. 2C). But, LC3B-II level was significantly increased by E64D + pepstatin A and was significantly reduced by 3-MA (Fig. 2C). This observation corroborates the well-established paradigm that LC3B-II level is indeed the surrogate of autophagic activity [12]. In contrast, CSE-induced LC3B-I, which is not a common phenomenon by other autophagy stimuli, was not dependent on autophagy; thus it appears to be a CS-specific phenomenon. We also did a pulse-chase study to further understand the kinetic change of LC3B. The cells were treated with/without CSE for 24 hrs, then CSE was removed and the level of LC3B was determined after 6 hrs. CSE significantly elevated both LC3B-I and II at 24 hrs (5^th^ lane, Fig. 2D). CSE removal for 6 hrs significantly reduced LC3B-I and II almost to the baseline (6^th^ lane, Fig. 2D), suggesting that this process is reversible. The decrease of LC3B-I (but not LC3B-II) after CSE removal was restored by 3-MA treatment (7^th^ lane, Fig. 2D), suggesting that autophagy was the main mechanism to clear up the increased LC3B protein. Enhanced autophagy flux even after CSE removal was demonstrated by the significantly elevated LC3B-II in CSE+ E+P treated cells (8^th^ Lane, Fig. 2D) as compared with E+P treated only cells (4^th^ Lane, Fig. 2D). Therefore, CSE regulates LC3B protein at both transcriptional and post-translational levels.

RETRACTED

**Figure 2:** CSE induced LC3B through at multiple levels. All western blot images were the representative image from at least three independent analyses, and Actin was use as a loading control. A) Time course of CSE induced LC3B and Nrf2. Cells were treated with 10% CSE. At each indicated time point, total protein was collected and subject to western blots analysis. B) CSE increased LC3B steady-state RNA. Cells were treated with 10% CSE. At each indicated time point, total RNA was collected and subject to Real-time PCR analysis. *: p<0.05, n = 5. C) CSE regulates LC3B-I and II at posttranslational levels. Cells were treated with 10% CSE for 24 hrs with either 3-MA (3MA) or lysozymal protease inhibitors-E64D and Pepstatin A (E+P). D) Pulse-chase study. Cells were treated with or without 10% CSE for 24 hrs. Then, CSE was removed and thoroughly washed. The cells were left alone (C) or treated with various inhibitors: cycloheximide (Cy), 3-MA (3MA) or E64D + Pepstatin A (E+P) for additional 6 hrs. Total protein was collected and subject to western blots analysis.

### 3. Nrf2 negatively regulated LC3B and autophagy, but independent of mTOR

Since CSE elevated both LC3B and Nrf2, we decided to examine the role of Nrf2 in the regulation of LC3B. We artificially increased Nrf2 level by overexpressing Nrf2. In these cells, LC3B-I and LC3B-II were significantly decreased (4^th^ lane, Fig. 3A) as compared to the mock-transfected cells (2th lane, Fig. 3A). Likewise, increased Nrf2 expression by siRNA knockdown of Keap1 (the cellular inhibitor of Nrf2) also repressed both LC3B-I and LC3B-II levels (6^th^ lane, Fig. 3B). Note: CSE appeared to significantly repress Keap1 expression (Fig. 3B). Conversely, Nrf2 knockdown further increased LC3B-I and II level by CSE (4^th^ lane, Fig. 3B), but not at the non-treatment condition (3^th^ lane, Fig. 3B). In addition, when both Nrf2 and Keap1 were knocked down, the levels of LC3B-I and II were restored to the similar level (8^th^ lane, Fig. 3B) as if Nrf2 was knocked down (4^th^ lane, Fig. 3B). Because LC3B-II is the hallmark of autophagy, we examined the impact of Nrf2 on autophagy. As shown in Fig. 3C, overexpression of Nrf2 (3C–e) or siRNA knockdown of Keap1 (3C–f) significantly repressed CSE induced autophagosomes. Fig. 3D shows the statistics of Fig. 3C from triplicates. Taken together, Nrf2 activation appears to repress CSE-induced LC3B-I and II as well as autophagosomes.

**Figure 3:** Nrf2 negatively regulate LC3B I and II. All western blot images were the representative image from at least three independent analyses, and Actin was use as a loading control. A) Effect of Nrf2 overexpression. Cells were transfected with Nrf2 plasmid (Nrf2) or empty vector (PCDNA3, or PC). 24 hrs later, cells were treated without (C) or with (CSE) 10% CSE for 24 hrs. B) Effect of siRNA knockdown of siNrf2 and/or Keap1. Cells were transfected with siRNA control (siC), siRNA against Nrf2 (siNrf2), siRNA against Keap1 (siKeap1), and siNrf2+siKeap1 (siN+K). 24 hrs later, cells were treated without (C) or with (CSE) 10% CSE for 24 hrs. C) Negative regulation of autophagosome by Nrf2. Cells stably transfected with GFP-LC3B were transfected with Nrf2 plasmid (Nrf2) or siRNA against Keap1 (siKeap1). Control was the mock-transfected cells. These cells were treated without (C) or with (CSE) 10% CSE for 24 hrs. Live images were recorded. “punctate dots” of GFP-LC3B were the indication of autophagosomes. D) Quantification of autophagosome (GFP-LC3B+ dots) was described in Materials and Methods. *, $: p<0.05, n = 3.

RETRACTED

Since mTOR is the master inhibitor of autophagy, we tested whether or not the repression of CSE-induced LC3B and autophagosome by Nrf2 was due to the activation of mTOR. CSE significantly repressed activated (phosphorylated) mTOR (Fig. 3A–B). The repression of mTOR activity was further corroborated by the decreased phosphorylated S6K (p-S6K) (Fig. 3A–B), a substrate of mTOR. However, neither Nrf2 overexpression nor Keap1 knockdown could restore the activations of both mTOR and S6K (Fig. 3A–B). Thus, mTOR is not the target of Nrf2 activation.

### 4. Increase of cellular GSH repressed CSE-induced LC3B and autophagosome but not mTOR

Nrf2 is a master regulator of antioxidant response partly through increasing the cellular reduced glutathione (GSH) level via activating several key GSH synthesizing enzymes [17]. Thus, we tested if the enhancement of GSH synthesis could recapitulate the effect of Nrf2 activation. Indeed, when supplementing the cells with N-acetylcysteine (NAC, a GSH precursor) or GSH itself, LC3B I and II were significantly repressed (Fig. 4B). In addition, these supplements repressed cellular ROS generation (Fig. 4A) and CSE-induced autophagosomes (Fig. 4C–D). Similar to Nrf2 activation, NAC or GSH was not able to restore the repressions of mTOR and S6K by CSE (Fig. 4B). Taken together, Nrf2 appears to repress CSE-induced LC3B level and autophagosomes through increasing the cellular antioxidants (e.g. GSH), thereby inhibiting CSE-induced oxidative stress. But, it has no effect on mTOR activity.

**Figure 4:** Antioxidant supplement repressed CSE-induced LC3B and autophagosome. A) Antioxidants neutralized CSE-induced cellular ROS. Cells were treated with 10% CSE or plus NAC (CSE+NAC) or GSH (CSE+GSH). Images were recorded 30 min after dye loading. Green fluorescence indicates generation of reactive oxygen species that oxidized the dye to emit fluorescence. B) Antioxidants downregulated CSE-induced LC3B. C) Antioxidants downregulated CSE-induced autophagosome. D) Quantification of autophagosome (GFP-LC3B+ dots) was described in Materials and Methods. *, $: p<0.05, n = 3.

### 5. P62 is another Nrf2-responsive gene and responsible for repressing CSE-induced LC3B and autophagosomes

To further understand the molecular mechanism underlying Nrf2-mediated LC3B repression, we searched for downstream effectors of Nrf2. HO-1, an Nrf2 downstream gene, has been shown to modulate CSE-induced LC3B [15]. We extended this finding by examining two additional well-known Nrf2 dependent genes- P62 [32] and NQO1 [33]. They are both elevated by CSE (2^nd^ lane, Fig. 5A–B). As shown in the previous study, single knockdown of Keap1 repressed LC3B-I and II (6^th^ lane, Fig. 3B) while double knockdown of Keap1 and Nrf2 could restore CSE-induced LC3B-I and II (8^th^ lane, Fig. 3B). Thus, we used the same strategy to determine whether or not either of these two proteins is the downstream effector of Nrf2. As shown in Fig. 5A, double knockdown of Keap1 and NQO1 couldn't restore the CSE-induced LC3B-I and II (8^th^ lane, Fig. 5A), and single knockdown of NQO1 also had no effect (4^th^ lane, Fig. 5A). In contrast, when both Keap1 and P62 were knocked down, CSE-induced LC3B-I and II were restored (8^th^ lane, Fig. 5B). To confirm this observation, we overexpressed P62 and it indeed repressed the elevations of LC3B-I and II induced by the increasing doses of CSE (6^th^-8^th^ lanes, Fig. 5C). Consistently, P62 overexpression also repressed CSE-induced autophagy (Fig. 5D–E). Thus, P62 appears to be the downstream effector of Nrf2 that mediates the repression of CSE-induced LC3B and autophagosomes.

RETRACTED

**Figure 5:** P62, but not NQO1, replicated Nrf2 phenotype. All western blot images were the representative image from at least three independent analyses, and Actin was use as a loading control. A) NQO1 knockdown couldn't rescue Keap1 knockdown. Cells were transfected with siRNA control (siC), siRNA against NQO1 (siN), siRNA against Keap1 (siK), and their combinations as indicated. 24 hrs later, cells were treated without or with 10% CSE for 24 hrs. Total proteins were collected for western blot analysis. B) P62 knockdown couldn't rescue Keap1 knockdown. Cells were transfected with siRNA control (siC), siRNA against P62 (siP), siRNA against Keap1 (siK), and their combinations as indicated. 24 hrs later, cells were treated without or with 10% CSE for 24 hrs. Total proteins were collected for western blot analysis. C) Effect of P62 overexpression. Cells were transfected with P62 plasmid (P62) or empty vector (PCDNA3, or PC). 24 hrs later, cells were treated without (C) or with (CSE) at increasing doses (8%, 10%, 12%) for 24 hrs. D) overexpression of P62 represses LC3B. Cells stably transfected with GFP-LC3B were transfected with P62 plasmid (P62) or empty vector (PCDNA3, or PC). These cells were treated without (C) or with (CSE) 10% CSE for 24 hrs. Live images were recorded. “punctate dots” of GFP-LC3B were the indication of autophagosomes. E) Quantification of autophagosome (GFP-LC3B+ dots) was described in Materials and Methods. *, $: p<0.05, n = 3.

## Discussion

CSE-induced autophagy appears to be different from the autophagy induced by conventional stimuli such as starvation. The conventional stimuli mostly increase the conversion from LC3B-I to LC3B-II, while the overall amount of LC3B appears to be constant. In contrast, CSE significantly increase the total amount of LC3B. The induction of LC3B-I appears to be much earlier than the increase of autophagy (as shown by the increase of LC3B-II). However, it is unclear whether CSE accelerates the autophagy biogenesis, which leads to more LC3B-I to LC3B-II conversion; or large amount of LC3B-I induced by CSE drives more LC3B-II conversion through a concentration-dependent passive mechanism. To investigate these possibilities, we blocked autophagy biogenesis using class III PI3K inhibitor 3-MA. There was no change in LC3B-I and II levels in untreated cells, but 3-MA significantly decreased LC3B-II in CSE-treated cells without affecting LC3B-I. In addition, when lysosomal protease activity was blocked, LC3B-II level was increased. These suggest that CSE did increase the autophagy biogenesis. It is surprising that, even without CSE treatment, LC3B was still recycled through lysozyme but is 3-MA insensitive. This process is perhaps mediated through other non-canonical autophagic pathways. In our pulse/chase study, we further demonstrate that CSE-induced LC3B is reversible. In the CSE-treated cells, autophagosome/lysosome-mediated post-translational degradation pathway plays an important role in maintaining LC3B level. The excessive LC3B-I was cleared within 6 hrs by autophagy. The increase of LC3B-I protein (also perhaps mRNA) by CS (or CSE) exposure appears not to be restricted in the lung epithelial cells [13], [15]. Similar observations have been made in other cell types such as macrophage [14], fibroblast [14], keratinocyte [34], endothelial cells [35], the follicle-associated epithelium and M-cells in peyer patches [36]. Thus, CS (or CSE) exposure is capable of modulating autophagy in various tissues of the body, and autophagy may play critical role in the pathogenesis of different CS-related illnesses.

RETRACTED

In addition to its traditional pro-survival role in the cellular response to stress conditions. excessive autophagy can also lead to cell death (type II) [37]. In the above-mentioned CS (or CSE) induced models, excessive autophagy appears to be largely associated with cellular damage and cell death. Chen ZH et, al. have elegantly demonstrated that LC3B, through interacting with Fas and Cav, regulates extrinsic apoptosis in CS-induced emphysema model [16]. However, CS (or CSE)-induced autophagy in immune related cells such as macrophage [14] and M cells [36] may have other functions. Indeed, autophagy has been well studied for its broad function in innate and adaptive immunity, including microbicidal activity [38], modulation of pattern recognition receptors [39], [40] and antigen presentation [41], [42]. Interestingly, microbials can also develop counter measures to hijack autophagic machinery for their own survival. For example, Staphylococcus aureus co-localizes with LC3B and its replication is dependent of autophagy [43]. In addition, Picornavirus (e.g. polio virus and rhinovirus) utilizes the surface of autophagosome as their replicating factory [44], [45]. Thus, increased autophagosomes by CS (or CSE) may facilitate the replication and growth of certain viruses or bacteria. To support this speculation, markedly enhanced rhinovirus replication has been demonstrated in the experimental rhinoviral infections on COPD patients [46] or on the epithelial cells derived from the airways of COPD patients [47]. Thus, further studies may be required to completely elucidate the interactions between virus and autophagosome in the context of virus-induced COPD exacerbation [48]–[50].

Another major distinction between CSE- and starvation-induced autophagy is the involvement of ROS and Nrf2 in the former. Nrf2 has been well established as the master regulator of cellular antioxidant pathway mainly via the activation of a battery of antioxidant gene expression [51]. The importance of Nrf2 in various lung diseases (e.g. acute lung injury, acute respiratory distress syndrome, asthma, COPD, lung cancer, infection etc.) has been extensively reported (reviewed in [51]). Although CSE induces both Nrf2 activation and autophagy, the interaction between these two pathways hasn't been clearly defined. The present study is the first report regarding their interactions in the CS-related models. Previous reports suggest that the lack of autophagy causes the accumulation of P62, which leads to persistent activation of Nrf2 via Keap1 (the cellular inhibitor of Nrf2) sequestration [22], [52]. Thus, Autophagy appears to act upstream to positively regulate Nrf2 activation. In the present study, we have found that the peak Nrf2 activation (6 hrs) occurred early than the peak of autophagy marker-LC3B-II level (24 hrs). The activation of Nrf2 either by overexpression or by Keap1 knockdown repressed LC3B-I and II and also decreased autophagosome number. Thus, our study indicates that Nrf2 acts upstream to negatively regulate CS-induced autophagy. Even more intriguingly, we found that P62 was the downstream effector of Nrf2 that repressed autophagy. Both studies are not entirely conflicting though, because a recent report suggests an Nrf2->p62->Nrf2 positive loop that regulates Nrf2 mediated anti-oxidant gene expression [32]. In their model of non-canonical Nrf2 activation, p62 is transcriptionally activated by Nrf2 via ARE site on its promoter; then the accumulated p62 sequesters Keap1 and subjects it to autophagic degradation, which leads to persistent Nrf2 activation [32]. However, this model has been established entirely in the non-pulmonary cell types such as HEK293, mouse embryonic fibroblasts, kidney cells and hepatocytes [22], [52]. Whether or not it also exists in pulmonary cells require further investigation. Another possibility is that CS-induced autophagy may be different from or be regulated differentially by the canonical autophagy. Previously, Kim HP et al. has demonstrated the protective role of HO-1 in repressing CSE-induced autophagy [15]. This observation supports our finding about the protective role of Nrf2 in CSE-induced autophagy because HO-1 is a classical Nrf2-dependent gene [51]. The present study identifies a second Nrf2-dependent gene product-P62 as another autophagy repressor. Thus, Nrf2 system is likely to play an indispensible role in regulating autophagy.

RETRACTED

Recently, Fujita, K et, al. indicates that Nrf2-P62 is required for TLR4 mediated aggresome-like induced structure (ALIS) formation [53]. This ALIS has autophagosome-like features such as LC3 positive and being degradable through lysosomal compartment. In their study, Nrf2-P62 appears to be a positive regulator of ALIS formation. However, classical autophagy inhibitors (3-MA and wortmannin) and siRNA knockdown of essential ATG (ATG5, ATG7) failed to prevent this process [53]. Thus, the formation of ALIS is different from the classical autophagy. Nonetheless, this study has reflects the complicated nature of Nrf2-P62 system in controlling a variety of LC3 associated cellular structures that warrant further study.

In summary, we have, for the first time, demonstrated that Nrf2 system negatively regulates CSE-induced LC3B expression and autophagosomes partly through the elevation of P62. The elucidation of this important interaction between Nrf2 systems and autophagy will advance our understanding of the pathogenic effect of CS-associated chronic airway diseases and reveal novel drug targets for the development of effective treatments.
